RETRACTED

# Glioma-Derived ADAM10 Induces Regulatory B Cells to Suppress CD8^+^ T Cells

**DOI:** 10.1371/journal.pone.0105350

**Published:** 2014-08-15

**Authors:** Zhuo-peng Ye, Hai-yong He, Hui Wang, Wen-sheng Li, Lun Luo, Zhen-chao Huang, Ying Guo

**Affiliations:** Department of neurosurgery, Third Affiliated Hospital of Sun Yat-sen University, Guangzhou, China; San Raffaele Scientific Institute, Italy

## Abstract

CD8^+^ T cells play an important role in the anti-tumor activities of the body. The dysfunction of CD8^+^ T cells in glioma is unclear. This study aims to elucidate the glioma cell-derived ADAM10 (A Disintegrin and metalloproteinase domain-containing protein 10) in the suppression of CD8^+^ effector T cells by the induction of regulatory B cells. In this study, glioma cells were isolated from surgically removed glioma tissue and stimulated by Phorbol myristate acetage (PMA) in the culture. The levels of ADAM10 in the culture were determined by enzyme-linked immunosorbent assay. Immune cells were assessed by flow cytometry. The results showed that the isolated glioma cells express ADAM10, which was markedly up regulated after stimulated with PMA. The glioma-derived ADAM10 induced activated B cells to differentiate into regulatory B cells, the later suppressed CD8^+^ T cell proliferation as well as the induced regulatory T cells, which also showed the immune suppressor effect on CD8^+^ effector T cell proliferation. In conclusion, glioma cells produce ADAM10 to induce Bregs; the latter suppresses CD8^+^ T cells and induces Tregs.

## Introduction

The tumor-tolerance plays an important role in the pathogenesis of glioma [1]. The induction of immune tolerance in a tumor environment is incompletely understood. The regulatory T cells (Tregs) and regulatory B cells (Bregs) are the major components of immune tolerance system in the body. The induction of Tregs and Bregs has been reported by many investigators. A number of molecules have been identified to have the ability to induce the immune regulatory cells; such as transforming growth factor (TGF)-β inducing Tregs was reported by Zheng et al [2] and Chen et al [3] in the early of 2000s. Liu et al indicate that fungus derived glucuronoxylomannan can induce Tregs [4]. Thus, it seems that the immune regulatory cells can be induced by multiple molecules. However, whether glioma is directly associated with the induction of immune regulatory cells is unclear.

In the studies of immune regulatory cells, investigators mainly focus on the characterization of Tregs. In recent years a number of publications show that Bregs are also important in the immune regulation in the body; such as van de Veen et al show that Bregs play a critical role in the restoration of immune tolerance in the process of specific immunotherapy [5]. Yet, the links between glioma and Bregs has not been elucidated.

RETRACTED

TGF-β is a major immune regulatory molecule in the induction of regulatory cells as well as fulfill the immune regulatory functions [6]. After synthesis, it exists as the precursor, the latent TGF-β. There is a latency associated peptide (LAP) attaches to the TGF-β complexes [7]. It is required to cleave such a LAP before the TGF-β gain the immune suppressor functions [7]. A large number of molecules are suggested to convert the latent TGF-β to the active form, TGF-β. Such as Chen et al indicate that integrin αvβ6 can convert the latent TGF-β to TGF-β [8]. ADAM10 has the proteolytic properties [9]. It can cleave proteins or peptides in a non-specific manner.

Based on published data that glioma cell contained ADAM10 [10], we hypothesized that glioma-derived ADAM10 can facilitate the induction of immune regulatory cells. Indeed, we observed that the glioma-derived ADAM10 induced Bregs, the latter has strong immune suppressor functions on inhibiting CD8^+^ T cells.

## Materials and Methods

### Reagents

The ADAM10 shRNA kit, antibodies of ADAM10 (A-3), TGF-β (D-12), LAP (T-17) and IgM (A-7) were purchased from Santa Cruz Biotech (Shanghai, China). ADAM10 ELISA kit, GI254023X, PMA, IL-2 and collagenase IV were purchased from Sigma Aldrich (Shanghai, China). The immune cell isolation kits were purchased from Miltenyi Biotech. CD40 was purchased from R&D Systems (Shanghai, China).

### Patients

Patients with glioma were recruited into the present study in our hospital from 2011 to 2013. The diagnosis and treatment were performed by their surgeons and pathologists. The using human tissue in the present study was approved by the Human Research Ethic Committee at Sun Yat-sen University. An informed, written consent was obtained from each human subject.

### Isolation of glioma cells

The glioma tissue was collected from the operation unit of our hospital. The tissue was cut into 2×2×2 mm pieces and incubated in the presence of collagenase IV (0.5 mg/ml) for 1 h at 37°C with mild stirring. The cells were filtered through a cell strainer. After washing, the cells were cultured in RPMI1640 medium supplemented with 10% fetal bovine serum (FBS), 100 U/ml penicillin, 0.1 mg/ml streptomycin and 2 mM L-glutamin. Immune cells (including CD3^+^ T cells and CD11c/b^+^ dendritic cells) were eliminated from the glioma cells by the magnetic cell sorting (MACS) with commercial reagent kits following the manufacturer's instructions.

### Naïve B cell isolation and culture

The peripheral blood mononuclear cells (PBMC) were isolated from the blood by gradient density centrifugation. CD19^+^ IL-7R^−^ CD45^+^ B cells were isolated from the PBMC by MACS using commercial reagent kits following the manufacturer's instructions. The cells were cultured with complete RPMI1640 medium in the presence of an anti-CD40 antibody at 10 ng/ml.

RETRACTED

### Generation of Bregs

Naïve B cells were cultured in the basal chambers of Transwells; the glioma cells were cultured in the inserts; the ratio of B cell and glioma cell was 5∶1. The medium was supplemented with anti-IgM (10 µg/ml), anti-CD40 (10 ng/ml) and PMA (20 ng/ml). The medium was changed in 3 days.

### Generation of Tregs by Bregs

Naïve CD4^+^ T cells were isolated from PBMC by MACS using a commercial reagent kit following the manufacturer's instructions. The T cells were cultured with Bregs at a ratio of 5∶1 in the presence of anti-IgM (10 µg/ml), anti-CD40 (10 ng/ml) and IL-2 (10 ng/ml). The medium was changed on day 3. The cells were collected on day 6. The Tregs were isolated with a Treg isolation kit following the manufacturer's instructions. The purity of the generated Tregs was greater than 90% as checked by flow cytometry.

### Enzyme-linked immunosorbent assay (ELISA)

Cytokine levels in culture medium were determined by ELISA with commercial reagent kits following the manufacturer's instructions.

### Quantitative real time RT-PCR (qRT-PCR)

The total RNA was extracted from the cells with the TRIzol reagents. The cDNA was synthesized using a reverse conversion reagent kit. The qPCR was carried out on a real time PCR device (MiniOpticon, Bio-Rad, Shanghai, China). The results were calculated with the 2^-ΔΔCt^ method. The data were normalized to percentage of the internal control gene, β-actin. The primers using in this study include: ADAM10: Forward, gggctgtgcagatcattcag; reverse, ctgggcaatcacagcttctc. β-actin: Forward, cgcaaagacctgtatgccaa; reverse, cacacagagtacttgcgctc.

### Western blotting

The proteins were separated by sodium dodecyl sulfate polyacrylamide gel electrophoresis (SDS-PAGE) and transferred onto nitrocellulose membranes; the membranes were blocked with 5% skim milk, incubated with the primary antibodies (0.1–0.5 µg/ml) and followed by the secondary antibodies (labeled with horseradish peroxidase). The immune blots on the membranes were developed by enhanced chemiluminescence (ECL). The results were recorded with X ray films. The integrated density of the immune blots was assessed by software PhotoShop (CS5).

### Flow cytometry

Cells were fixed with 2% paraformaldehyde (mixed with 0.1% Triton X-100 in case the intracellular staining) for 1 h at room temperature. The cells were blocked by incubation with 1% BSA followed by incubation with antibodies (labeled with fluorescence). After washing, the cells were analyzed by flow cytometry. To assess the CD8^+^ effector T cell proliferation, CD8^+^ CD25^−^ T cells were isolated from the peripheral blood mononuclear cells (PBMC), labeled with CFSE (carboxyfluorescein diacetate, succinimidyl ester; 5 µM), cultured with or without the presence of Tregs or Bregs for 3 days in the presence of anti-CD3/CD28 antibodies and PMA (20 ng/ml). The proliferation of the CD8+ T cells was assessed with a flow cytometer.

RETRACTED

### Over expression of ADAM10 in glioma cells

The genomic DNA was extracted from the isolated glioma cells. The ADAM10 gene was amplified by PCR. The PCR products were sequenced first and confirmed, and cloned into the pTZ57R/T vector and transformed into *E. coli*. The vectors of ADAM10 gene were subcloned into the pcDNA3 plasmid and transformed into competent *E. coli* by the heat shock method. The plasmid was then purified using a plasmid extraction kit according to the manufacturer's instructions. The presence of the ADAM10 gene was confirmed by sequencing. The glioma cells were transfected with the constructed ADAM10 plasmids using a transfection reagent kit according to the manufacturer's instructions.

### ADAM10 gene silence in glioma cells

Glioma cells were treated with shRNA reagent of ADAM10 following the manufacturer's instructions. The gene knockdown effect was assessed by Western blotting, which lasted at least 4 weeks.

### Statistics

The data were presented as mean ± SD. Differences between groups were determined by ANOVA. P<0.05 was set as a significant criterion.

## Results

### Increases in ADAM10 expression in Glioma cells upon activation

The glioma cells were isolated from the surgically removed glioma tissue (low grade: n = 3; high grade: n = 3) and stimulated by PMA in the culture for 48 h. The cells were analyzed by qRT-PCR and Western blotting. The results showed that low levels of ADAM10 were detected in the low and high grade glioma cells cultured in medium alone. Exposure to PMA markedly increased the expression of ADAM10 in the glioma cells of both low grade and high grade in a PMA dose-dependent manner (Fig. 1A, 1B). To elucidate if the ADAM10 could be released out the glioma cells, we measured the levels of ADAM10 in the culture supernatant by ELISA. The results showed that the levels of ADAM10 was below the detectable levels while cultured in medium alone. Exposure to PMA significantly increased the levels of ADAM10 in the culture supernatant (Fig. 1C). The results indicate that both low grade and high grade glioma cells express ADAM10 that can be up regulated upon activation, which can be released to the microenvironment.

RETRACTED

**Figure 1:** Activation increases ADAM10 expression in glioma cells. Human glioma cells (low grade: n = 3; high grade: n = 3) were cultured in the presence of PMA for 48 h. The doses of PMA are denoted in each subpanel. The cell extracts were analyzed. A, the immune blots indicate the protein levels in the cellular extracts. The bars below the blots indicate the integrated density of the immune blots. B, the bars indicate the levels of mRNA. C, the bars indicate the protein levels in the culture supernatant (by ELISA). The data of bars are presented as mean ± SD. *, p<0.01, compared with dose “0”. The data shown is a representative from 3 separate experiments.

### Glioma-derived ADAM10 induces Bregs

We next observed that the glioma-derived ADAM10 induced Bregs. Naïve B cells were isolated from peripheral blood mononuclear cells (PBMC) and cultured together with the isolated glioma cells in Transwell system or cultured alone. After exposure to PMA in the culture, the cells were analyzed by Western blotting. The results showed that, when cultured alone, PMA increased LAP (Fig. 2A), but not TGF-β (Fig. 2B), expression in B cells. The presence of glioma cells and PMA in the culture induced TGF-β in the B cells (Fig. 2B). Since TGF-β is one of the key molecules of immune regulatory cells [11], the results indicate that the glioma-derived ADAM10 can convert naïve B cells to Bregs. To strengthen the results, we added the inhibitor of ADAM10 in the culture. The Breg conversion was abolished (Fig. 2B). Over expression of ADAM10 (Fig. 2C) in the glioma cells also induced Breg (Fig. 2B). The knockdown of ADAM10 gene (Fig. 2D) in glioma cells disabled the induction of Bregs (Fig. 2B).

**Figure 2:** Glioma induces Breg. A, naïve B cells were treated with PMA at graded doses in the culture for 48 h. The cells were collected; the cellular extracts were analyzed by Western blotting. The immune blots indicate the protein levels of latency associated peptide (LAP). B, naïve B cells were cultured with glioma cells in Transwells at a ratio of 1∶1 in the presence of PMA (20 ng/ml) for 6 days. The additional treatment is denoted on the X axis. The immune blots indicate the protein levels of TGF-β in the B cell extracts. No glioma: B cells alone. Glioma: B cells were cultured with glioma cells. #, ADAM10 inhibitor (GI254023X; 5 µM) was added to the culture. O-exp (O-exp-con): The glioma cells were transfected with ADAM10 plasmid (the “con” indicates an empty plasmid). ADAM10-null: ADAM10 gene was knocked down in the glioma cells by transducing with ADAM10 shRNA. cshRNA: The glioma cells were transduced with control shRNA. C, the immune blots indicate the ADAM10 over expression (O-exp) results in glioma cells. D, the immune blots indicate the results of ADAM10 gene knockdown in glioma cells. The bars of A and B indicate the integrated density of the immune blots measured by ImageJ. *, p<0.01, compared with dose “0” (A), or saline (B). The data shown is a representative from 3 independent experiments.

RETRACTED

### Glioma-converted Bregs suppress CD8^+^ T cells

We assessed the immune suppressor functions of the glioma-converted Bregs. CD8^+^ T cells were isolated from PBMC, labeled with CFSE, and cultured with the Bregs at a ratio of 1∶5 (Breg:T cell) for 3 days in the presence of anti-CD3/CD28 and PMA. As shown by flow cytometry data, exposure to anti-CD3/CD28 markedly induced CD8^+^ T cell proliferation (Fig. 3A, 3B, 3E), which was abolished by the Bregs (Fig. 3C, 3E). The results indicate that the Bregs have the ability to suppress CD8^+^ T cell proliferation. Since the expression of TGF-β was detected in the Bregs, we inferred that the immune suppression was mediated by TGF-β. To test the inference, we added a neutralizing anti-TGF-β antibody to the culture. The suppression of CD8^+^ T cell proliferation was abolished (Fig. 3D, 3E). The results confirm that the immune suppression on CD8^+^ T cells by Bregs is mediated by TGF-β. To strengthen the results, we measured the levels of perforin, one of the major cytotoxic mediators of CD8^+^ T cells, in the culture supernatant. The results showed that the perforin could be detected in the supernatant and could be altered in parallel with the changes of CD8+ T cell proliferation (Fig. 3F).

**Figure 3:** Glioma-induced Bregs suppress CD8^+^ T cell activities. Bregs were prepared as described in Fig. 2. CD8^+^ CD25^−^ T cells were isolated from PBMC, labeled with CFSE, and cultured with Bregs at a ratio of 1∶5 (Breg:T cell) for 3 days in the presence of anti-CD3/CD28 antibodies and PMA (20 ng/ml) or an anti-TGF-β antibody (50 ng/ml). A–D, the cells were analyzed by flow cytometry. The treatment is denoted above each subpanel. The histograms indicate the frequency of proliferated CD8^+^ T cells which were summarized in E. F, the bars indicate the levels of perforin in the culture supernatant (by ELISA). The data in E and F are presented as mean ± SD. *, p<0.01, compared with group A. The data shown is a representative from 3 separate experiments.

### Glioma-induced Bregs induce Tregs

Based on the published data that exposure to TGF-β can induce Tregs, we hypothesize that the glioma-induced Bregs can induce Tregs. To test the hypothesis, we isolated naïve CD4^+^ T cells from PBMC and cultured with the Bregs in the presence of PMA for 6 days. The cells were analyzed by flow cytometry. The results showed that about 60% T cells were converted to Tregs based on the expression of TGF-β (Fig. 4A). No appreciable Tregs were converted by naïve B cells (Fig. 4B). The data confirm that the glioma-converted Bregs can induce Tregs. To test the immune suppression of the induced Tregs, we cultured the Tregs with CD4^+^ CD25^−^ effector T cells (labeled with CFSE) in the presence of anti-CD3/CD28 for 3 days. Indeed, the induced Tregs showed strong immune suppressor functions (Fig. 4D–F, 4H) which was abolished in the presence of a neutralizing antibody in the culture (Fig. 4G, 4H).

RETRACTED

**Figure 4:** Immune suppressor assessment of the induced Tregs. A–B, Bregs (A) or naïve B cells (B) and naïve CD8^+^ T cells were cultured in the presence of PMA and IL-2 for 6 days. The dot plots indicate the frequency of Tregs. C, the bars indicate the summarized frequency of Tregs in A and B. D–G, the Tregs in A were isolated by MACS and cultured with effector CD8^+^ T cells (labeled with CFSE. The additional treatment was denoted above each subpanel. The histograms indicate the frequency of proliferated effector T cells. H, the bars indicate the summarized data of D–G. The data of bars are presented as mean ± SD. *, p<0.01, compared with Breg group (C), or with group D (H). The data shown is a representative from 3 separate experiments.

## Discussion

The present data show that glioma cells produce ADAM10 upon activation. The ADAM10 can induce Bregs by converting LAP to TGF-β in the B cells. The Bregs have immune suppressor functions by showing the suppression ability on CD8^+^ T cell activities. The Bregs also have the ability to induce Tregs. Immune regulatory cells play an important role in tumor cell escaping from the immune surveillance. Inhibition of Tregs has been suggested to inhibit tumor growth [12].

ADAM10 has the proteolytic enzyme properties [9], [10]. Cumulative reports indicate that ADAM10 is involved in the immune regulation. Moller et al reports that ADAM10 cleaves the T cell immunoglobulin and mucin domain 3 (Tim-3) to regulate T cell activities [13]. Hoffmann et al indicate that ADAM10 cleaves CD84 from the surface of platelet to modulate the interaction between immune cells and platelet [14]. Our data are in line with those studies by showing that ADAM10 can cleave the LAP to activate TGF-β in B cells. It is reported that activation can induce the latent TGF-β in B cells. The latent TGF-β does not have immune suppressive functions until activated. The present data indicate that glioma-derived ADAM10 has such an ability to convert the latent TGF-β to TGF-β in the B cells. The B cells thus have the immune suppressive functions. Supportive data have been reported in other regulatory cell generation systems. Wang et al indicate that glycoprotein-A repetitions predominant protein can cleave the LAP from the TGF-β complex to activate TGF-β [15]. Our data are in line with those reports. However, these Bregs suppress CD8^+^ T cells; the latter is an important anti-tumor cell population.

RETRACTED

The data also show that the glioma-induced Bregs have the ability to induce Tregs. Although the data are relative new, supportive evidence was obtained in the present study. The induction of Tregs by the glioma-induced Bregs is mediated by TGF-β since the induction can be blocked by the presence of a neutralizing anti-TGF-β antibody.

In summary, the present data indicate that glioma can induce Bregs by releasing ADAM10. The Bregs can suppress CD8^+^ T cell activities as well as induce Tregs.
